RETRACTED

# Regional effects of the renewable energy components on CO_2_ emissions of Asia-Pacific countries

**DOI:** 10.1371/journal.pone.0256542

**Published:** 2021-10-13

**Authors:** Man-Wen Tian, Shu-Rong Yan, Mohsen Khezri, Muhaamad Sharif Karimi, Mahnaz Mamghaderi, Yousaf Ali Khan

**Affiliations:** 1 National Key project Laboratory, Jiangxi University of Engineering, Xinyu, China; 2 Faculty of Economics and Social Sciences, Bu-Ali Sina University, Hamedan, Iran; 3 Department of Economics, University of Kurdistan, Hewler, Kurdistan Region of Iraq; 4 Department of Economics, Razi University, Kermanshah, Iran; 5 Department of Mathematics and Statistics, Hazara University, Mansehra, Pakistan; Universiti Teknologi Petronas, MALAYSIA

## Abstract

This paper utilizes spatial econometric reenactments to examine the geographic effects of different types of environmentally friendly power on corban discharges. The example covers 31 nations in the Asia-Pacific district during the time frame 2000 to 2018. The spatial connection in the model was affirmed by symptomatic testing, and the spatial Durbin model was picked as the last model. Results show that Gross domestic product per capita, receptiveness to business sectors, unfamiliar direct venture, energy force, and urbanization critically affect CO_2_ emanations. In correlation, just wind and sunlight-based energy have added to a generous abatement in ozone harming substance emanations in nations over the long run. In contrast, hydropower, bioenergy, and geothermal energy discoveries have been irrelevant. A cross-sectional examination worldview delineated that nations with more elevated sunlight-based energy yield have higher CO_2_ outflows, while nations with lower levels have lower CO_2_ emanations. The presence of spatial impacts in the model gave off an impression of the negative consequences for homegrown CO_2_ outflows of Gross domestic product per capita and exchange transparency of adjoining nations. Furthermore, energy power and higher creation of sustainable power in adjoining nations will prompt lower homegrown CO_2_ outflows.

## 1. Introduction

Environmental change identified with ozone-depleting substance emanations, CO_2_ outflows from energy utilization, represents a colossal extent of all GHG discharges throughout many years, as per Paramati et al. [1]. The consumption of petroleum products, for example, coal, oil and flammable gas, represents most of fossil fuel byproducts, representing over 80% of worldwide energy interest, and the essential driver of a dangerous atmospheric deviation is the emanation of ozone harming substances, of which 72% is carbon dioxide (CO_2_). Rising CO_2_ contamination is likewise a worldwide test, and worldwide environmental change has caused worldwide feelings of dread.

RETRACTED

Expanding parts of worldwide energy creation frameworks and energy framework upgrades and changing to cleaner energy. For example, sustainable power can adjust CO_2_ emanations levels and lead to outflow decreases. The goal of an environmentally friendly power, which has arisen as a compelling option in contrast to petroleum products and is generally acknowledged as a critical factor for an Earth-wide temperature boost, is one arrangement. Then again, by supplanting petroleum products, environmentally friendly power is an ideal hotspot for a cleaner energy utilization structure, bringing about fewer CO_2_ outflows in exact examinations (Bilgili et al. [2]; Moutinho and Robaina [3]; Kahia et al. [4]; Bekun et al. [5]). Likewise, various investigations have featured the peripheral or even certain effect of environmentally friendly power use on the dispersion of CO_2_ outflows, particularly in low-medium-pay nations. Apergis and Payne [6] have demonstrated that sustainable power isn’t assisting with diminishing CO_2_ outflows in the 19 created and agricultural nations for the time being. Farhani [7] exhibits only single-directional causality in the present moment from efficient power energy utilization to CO_2_ emanations, and the outcomes are negligible over the long skyline. The observational exploration of Ben Jebli and Youssef [8] for 5 North African nations found that utilization of efficient power energy brings about more CO_2_ discharges. Sustainable power utilization triggers CO_2_ contamination in low-pay countries, in view of Nguyen and Kakinaka [9]. As of late, Saidi and Omri [10] have indicated that spotless energy consumption in certain nations diminishes CO_2_ outflows, yet this raises CO_2_ discharges in the Netherlands and South Korea. Ben Jebli et al. [11] determined that environmentally friendly power utilization in higher-pay nations diminishes CO_2_ emanations, so the results for low-center pay nations were good for nothing.

The impacts of different parts of sustainable power regarding an expansive example of nations and the likely spatial impacts between model factors have been disregarded in the trial writing up until this point, despite the clashing discoveries acquired in certain investigations. A more intensive glance at the impact of all environmentally friendly power parts on CO_2_ outflows will likewise permit policymakers to assess environmentally friendly power strategy structures, considering the estimation of environmentally friendly power development in accomplishing the feasible improvement of nations. In this sense, the vital goal of the exploration is to dissect the potential impacts of environmentally friendly power parts on CO_2_ emanations for a wide example of 31 nations, considering the provincial varieties between locales in the Asia-Pacific district for the years 2000–2018.

RETRACTED

Subsequently, this exploration tries to research the impact of sustainable power sources on CO_2_ emanations, just as to break down the effect of inflows of the unfamiliar direct venture (FDI) on CO_2_ discharges. In past investigations on the part of FDI in CO_2_ emanations, two restricting thoughts have been proposed. The initially proposed FDI inflow is an instance of the more serious level of research and development uses, and the two of them improve monetary advancement in host nations, which thus will expand CO_2_ outflows by raising energy interest (Feridun et al. [12]; Lau et al. [13]; Seker et al. [14]; Tang and Tan [15]). Second, FDI is a significant wellspring of cutting-edge innovation financing and change and is considered (Tamazian et al. [16]; Alam et al. [17]; Paramati et al. [18]). Considering the differentiating sees among analysts, the connection among FDI and CO_2_ outflows, new and more nitty-gritty econometric models and a more extensive and more intensive example of the nations under survey, which is underscored in this investigation, should be analyzed.

This proposition is separated from past investigations on the exploration subject by two significant attributes and prompts making up for the shortcoming in writing. To begin with, while some past examinations have explored the connection between sustainable power and CO_2_ emanations. They focused distinctly on one file of absolute inexhaustible utilization among nations where all types of environmentally friendly power, including wind, sun oriented, hydropower, bioenergy and geothermal, are remembered for this exploration. Second, to the most amazing aspect of our agreement, no trials utilizing spatial econometric methodologies have examined the job of environmentally friendly power energy in CO_2_ emanations. Board information examination of past investigations can be isolated into two classes: first, the powerful OLS assessor was utilized to assess the effect of sustainable power use on CO_2_ discharges, for example, GMM, FMOLS, PMG and DOLS (for reference, see Apergis and Payne [19]; Shafiei and Salim [20]; Dogan [21] and Seker [14]. Besides, the ecological supportability of close-by nations would be impacted by the key nation’s development and environment. A performing country will likewise affect its adjoining nations and locales. As ordinary board econometric techniques, due to evading spatial similitudes and neglecting to get the circuitous (neighborhood impacts) and spatial overflow effect of monetary development on CO_2_ discharges, add to slanted evaluations, with the end goal that the utilization of spatial econometric models is more compelling and beneficial (Meng et al. [22]; You and Lv [23]. Thirdly, it is critical to investigate the connection between CO_2_ outflows and the utilization of sustainable power in Asia-Pacific nations, particularly in battling an unnatural weather change. The remainder of this examination is coordinated as follows. The information and econometric techniques are recorded in Section 2. The logical results are introduced in Section 3, and their belongings are examined. Section 4 closures the paper and offers suggestions for strategy.

RETRACTED

## 2. Brief literature review

We discovered shifting connections between environmentally friendly power, financial turn of events, CO_2_ emanations, and different factors in writing. This variety in discovery seems to rely upon the choice to test, various techniques for investigation, the factors utilized in the examination, various nations and districts, and, as indicated by writing, for instance, the investigation time frame (Abulfotuh [24]; Bilgili et al. [2]; Dong et al. [25]). In Asia-Pacific nations, practical energy (for example, hydropower, sun-powered, wind, geothermal and biomass) has emerged as an effective option in contrast to petroleum products (for example, coal, petrol and flammable gas) with developing inquiries concerning the ecological and wellbeing results of CO_2_ discharges. Thinking about the above setting, a more precise comprehension of the nexus between CO_2_ discharges and efficient power energy is particularly applicable.

Menyah and Wolde-Rufael [26] exhibit that the utilization of environmentally friendly power was not the clarification for CO_2_ discharges from Granger. CO_2_ outflows were the purpose behind environmentally friendly power utilization from Granger. Vaona [27], then again, contends that higher utilization of non-sustainable power invigorates monetary development; however, that higher creation brings down the development pace of non-sustainable power utilization, likely because of higher energy effectiveness. Likewise, Farhani [7] explores the relationship between MENA nations’ utilization of sustainable power and CO_2_ discharges. Its discoveries propose a single direction causality from environmentally friendly power use to CO_2_ outflows. There is a single direction causality stretching out from CO_2_ emanations to extended haul utilization of sustainable power. This is similar to Apergis and Payne [19] or to seven nations in Focal America that distinguish a bi-directional causal relationship between’s the utilization of efficient power energy and CO_2_ outflows.

RETRACTED

To dissect causality between environmentally friendly power use, CO_2_ discharges and monetary development, Saidi and Mbarek [28] expressed that environmentally friendly power utilization diminishes CO_2_ emanations. They utilized changed common least square, unique conventional least square, and Granger causality measures. Paramati et al. (2016) uncover that in 20 creating market economies, environmentally friendly power use and per capita Gross domestic product assume a significant part in lessening per capita CO_2_ discharges. Besides, Balsalobre-Lorente and Shahbaz [29] attest that CO_2_ discharges are restricted by sustainable power use. Furthermore, Ito (2017) utilized GMM to characterize the connections between CO_2_ discharges and environmentally friendly power use and monetary development for a board of 42 created nations and found that environmentally friendly power use adds to emanations decreases and financial development rises. Ben Jebli and Youssef [8] look at sustainable power and horticulture in decreasing CO_2_ outflows in North African nations through Granger causality tests over 1980–2011. The studies show a unidirectional causality going from Gross domestic product to environmentally friendly power utilization and momentary farming from environmentally friendly power utilization. Besides, unidirectional causality streams from sustainable powers to agribusiness and, in the long haul, from contamination. Likewise, it is recommended that North African nations uphold the utilization of efficient power energy and, specifically, practical environmentally friendly power, for example, sun-oriented or wind energy, as this increments agrarian profitability and assists with handling an Earth-wide temperature boost.

Belaid and Youssef [30] likewise utilize the Granger causality procedure of the vector mistake remedy model (VECM) and propose that sustainable power use has a valuable natural impact in the long haul. Likewise, Bhattacharya et al. [31]. Uncover that environmentally friendly power utilization development adversely affects CO_2_ emanations for a board of 85 overall created and creating economies. They utilize the summed up framework strategy for minutes (GMM) and conventional least-squares completely altered (FMOLS).

Also, Zoundi [32] investigates the impact of sustainable power on natural demolition in 25 chose African nations and delineates that environmentally friendly power negatively affects CO_2_ emanations. Likewise, the board cointegration system utilized by Liu et al. [33] to analyze the nexus between sustainable power, farming and CO_2_ emanations, the discoveries uncovered that utilization of environmentally friendly power assumes a negative part in outflows, even though there is no causality between sustainable power and development in agribusiness. Then again, on account of Malaysia, Bekhet and Othman [34] explore dynamic collaboration between environmentally friendly power and CO_2_ emanations and Gross domestic product for the time frame from 1971 to 2015 and utilize VECM Granger techniques for causality, they found that sustainable power adversely affects CO_2_ discharges. The heading of causality runs from CO_2_ outflows to environmentally friendly power. More recently, Chen t al. [35] explores the relationship between China’s CO_2_ emissions, economic development, renewable and nonrenewable energy and international exchange and illustrates that renewable Energy and CO_2_ emissions are decreased. In addition, Dong et al. [36] demonstrate the impact of renewable energy consumption on CO_2_ emissions and suggest that increased renewable energy consumption will result in lower emissions of CO_2_. For the case of India, Kang et al. [37] investigated the relationships between CO_2_ emissions, renewable (wind, solar, or hydro) and nonrenewable energy sources (hydroelectric and coal) and economic development, applied a three-variable VAR model during 1965Q1-2015Q4, demonstrated that the proportion of renewable energy in total energy usage has risen over time in India. They proposed a complex relationship. In a more recent study, Ben Jebli et al. [11] used the Generalized Moment Method (GMM) framework to analyze the relationship between renewable energy, CO_2_ emissions, and economic development for 102 countries over the period 1990–2015. They found that renewable energy consumption positively affects all countries’ added manufacturing and service values. In addition, renewable energy consumption in all countries, except for lower-middle-income countries, gives rise to reduced CO_2_ emissions. In addition, Saidi and Omri [10] use the Completely Updated OLS (FMOLS) and the vector error correction model to analyze the relationship between CO_2_ pollution, clean energy and nuclear energy consumption in 15 OECD countries (VECM). Their findings suggest that developments in clean energies and nuclear energy in OECD countries decrease CO_2_ emissions. The results of the VECM process show that nuclear and renewable energy sources reduce CO_2_ emissions in the long run.

RETRACTED

## 3. Methodology and data

### 3.1. Empirical model

In this study, the effects of CO_2_ emission determinants focusing on renewable energy components are studied using spatial econometric models. An expanded version of Acheampong et al. (2020) follows the general shape of the carbon pollution rate model that we plan to analyze experimentally in this study. The logarithm of carbon emissions in this analysis (*lnCO*_2_) is considered as a function of the logarithm of GDP per capita (*lnGDPP*), the squared form of GDP per capita (*lnGDPP*^2^), energy intensity (*lnENER*), trade openness (*lnOPE*), urbanization (*lnURB*), and Foreign direct investment (*FDI*) The linear form of Eq 1 is used for experimental estimation:

$$ln{CO}_{2it}=\beta_{1}+\beta_{2}ln{GDPP}_{it}+\beta_{3}ln{GDPP}_{it}^{2}+\beta_{4}ln{ENER}_{it}+\beta_{5}ln{OPE}_{it}+\beta_{6}ln{URB}_{it}+\beta_{7}{FDI}_{it}+\beta_{8}{RENEW}_{it}+c_{i}\left(optional\right)+\alpha_{t}\left(optional\right)+\upsilon_{it}$$ (1)

Variables of urbanization and energy usage (Çelik and Deniz [38]; Epule et al. [39]; Bing et al. [40]; Chakravarty and Tavoni [41]), and exchange transparency are also used as explanatory variables for CO_2_ emissions (see Solarin et al. [42]). The relationship between economic development and environmental quality is shown by the theory of Environmental Kuznets (EKC). According to this theory, if the pace of economic development rises, the efficiency of the atmosphere first decreases and then improves (Lee et al. [43]; Grossman and Krueger [44]). According to the EKC hypothesis, the efficiency of the atmosphere is an inverted U-shaped related to the rise in economic growth. Thus the coefficient of the squared form of GDP per capita in the pollution equation CO_2_ must be negative.

This research explores the effect on CO_2_ emissions of renewable energy components domestically and in neighboring countries to evaluate the spatial dependency between observations. Different spatial models were calculated for this reason. A spatial panel model can have a lagged dependent variable or adopt a spatially autoregressive mechanism in the error word, according to Anselin et al. [45]. The spatial Durbin model, which involves spatially lagged model-independent variables, was also implemented by LeSage and Pace [46]. The basic formula of each of the three models is presented below. The model of spatial lag, the model of spatial fault, and the spatial model of Durbin are formulated as follows:

$$y_{it}=\lambda \sum_{j=1}^{N}w_{ij}y_{jt}+\varphi +x_{it}\beta +c_{i}\left(optional\right)+\alpha_{t}\left(optional\right)+\upsilon_{it}$$ (2)

$$y_{it}=\lambda \sum_{j=1}^{N}w_{ij}y_{jt}+\varphi +x_{it}\beta +c_{i}\left(optional\right)+\alpha_{t}\left(optional\right)+u_{it}$$ (3)

$$y_{it}=\lambda \sum_{j=1}^{N}w_{ij}y_{jt}+\varphi +x_{it}\beta +\sum_{j=1}^{N}w_{ij}x_{ijt}\theta +c_{i}\left(optional\right)+\alpha_{t}\left(optional\right)+\upsilon_{it}$$ (4)

where *y*_*it*_ is the dependent variable for cross-sectional unit *i* = 1, …, *N* at time *t* = 1, …, *T*. *x*_*it*_ is a 1 × K vector of exogenous variables, and *β* a *K* × 1 vector of parameters. The variable $\sum_{j=1}^{N}w_{ij}y_{jt}$ denotes the interaction effect of the dependent variables *y*_*jt*_ in neighboring units on the dependent variable *y*_*it*_. *w*_*ij*_ is the *i*, *j* − *th* element of a prespecified nonnegative *N* × *N* spatial weights matrix *w*. λ is the response parameter of these endogenous interaction effects. *υ*_*it*_ is an independently and identically distributed error term. *c*_*i*_ denotes a spatial specific effect and *α*_*t*_ a time-period-specific effect. In the spatial error model, the error term of unit *i*, $u_{it}=\rho \sum_{j=1}^{N}w_{ij}u_{jt}+\upsilon_{it}$, is taken to depend on the error terms of neighboring units j according to the spatial weights matrix W and an idiosyncratic component *υ*_*it*_. LeSage and pace [46] also recommend considering the spatial Durbin model. This model extends the spatial lag model with spatially lagged independent variables where *θ* is a *K* × 1 vector of parameters.

RETRACTED

### 3.2 Data

This study investigates the effects of CO_2_ emission determinants using data from 31 Asia-Pacific countries from 2000 to 2018. Fig 1 shows the amount of per capita renewable energy capacity in countries in simple terms. All variables are in the form of logarithms that can be interpreted as elasticity. For renewable energy components, the logarithm value plus one is calculated since the value of the variables in some years is zero. A summary of the constructed variables is presented in Table 1, whereas Table 2 summarizes the summary statistics of the data. The CO_2_ emissions per capita and per capita renewable energy emissions in the countries under study are shown in Fig 1. This figure illuminates that the spatial interaction between CO_2_ emissions tends to be regionally integrated into different countries. But to analyze this problem in more detailed detail in Fig 2, we need to remember Moran’s I statistics.

**Fig 1:** Corban emissions per capita and renewable energy per capita.

**Fig 2:** Moran’s I statistics for CO_2_ emissions per capita and renewable energy per capita.

**Table 1:** Variables constructed.

Variable	Variable constructed	Source
*lCO*_2*it*_	*lCO*_2*it*_ = *log*(*CO*_2*it*_) *CO*_2*it*_ = *CO*_2_ Emissions (metric tons per capita) in the country *i* in period *t*	SDG
*lRENEW*_*it*_	*lRENEW*_*it*_ = *log*(*RENEW*_*it*_) *RENEW*_*it*_ = Renewable energy per capita	SDG
*lHYD*_*it*_	*lHYD*_*it*_ = *log*(1 + *HYD*_*it*_) *HYD*_*it*_ = Hydropower Energy per capita	SDG
*lSOL*_*it*_	*lSOL*_*it*_ = *log*(1 + *SOL*_*it*_) *SOL*_*it*_ = Solar Energy per capita	SDG
*lWIN*_*it*_	*lWIN*_*it*_ = *log*(1 + *WIN*_*it*_) *WIN*_*it*_ = Wind Energy per capita	SDG
*lBIO*_*it*_	*lBIO*_*it*_ = *log*(1 + *BIO*_*it*_) *BIO*_*it*_ = Bioenergy Energy per capita	SDG
*lGEO*_*it*_	*lGEO*_*it*_ = *log*(1 + *GEO*_*it*_) *GEO*_*it*_ = Geothermal Energy per capita	SDG
*lGDP*_*it*_	*lGDP*_*it*_ = *log*(*GDPP*_*it*_) *GDP*_*it*_ = GDP per capita in 2010 prices$ in the country *i* in period *t*	WDI
*FDI*_*it*_	*FDI*_*it*_ = Foreign direct investment, net inflows (as a percentage of GDP)	WDI
*lURB*_*it*_	*lURB*_*it*_ = log(*URB*_*it*_) *URB*_*it*_ = Urban population (as a percentage of total population)	WDI
*lOPE*_*it*_	*lOPE*_*it*_ = *log*(*OPE*_*it*_) *OPE*_*it*_ = Trade Openness (total exports and imports as a percentage of GDP(	WDI
*lENER*_*it*_	*lENER*_*it*_ = log(*ENER*_*it*_) *ENER*_*it*_ = Energy intensity (energy use as a percentage of GDP)	SDG

WDI: World Development Indicator; https://datacatalog.worldbank.org/dataset/world-development-indicators.

RETRACTED

SDG: The Asia-Pacific SDG Gateway; https://data.unescap.org/.

IMF: International Monetary Fund; https://data.imf.org/.

**Table 2:** Summary statistics of the variables over the years 2000–2018.

Variable	Mean	Median	Maximum	Minimum	Std. Dev.	Observations
*lCO*_2*it*_	0.88	1.15	2.97	-2.34	1.37	558
*lRENEW*_*it*_	4.28	4.26	7.37	0	1.77	558
*lHYD*_*it*_	3.99	4.14	7.21	0	1.94	558
*lSOL*_*it*_	0.58	0.03	5.86	0	1.15	558
*lWIN*_*it*_	0.78	0.01	5.28	0	1.33	558
*lBIO*_*it*_	1.04	0.4	4.03	0	1.28	558
*lGEO*_*it*_	0.43	0	5.33	0	1.09	558
*lGDP*_*it*_	8.29	8.13	10.96	5.84	1.39	558
*FDI*_*it*_	4.37	2.63	55.08	-37.15	6.47	558
*lURB*_*it*_	3.86	3.94	4.61	2.6	0.49	558
*lOPE*_*it*_	4.16	4.16	6.08	-1.79	0.94	558
*lENER*_*it*_	1.75	1.7	3.53	0.69	0.49	558

### 3.3 Ethics statement

This article does not contain any studies with human participants or animals performed by any of the authors.

The two dimensions of Fig 2 correspond to geographic observations and their details on spatial lag. A positive Moran I represents the spatial accumulation of identical values in Quadrants I and III across the section presented, while a negative value represents the spatial accumulation of non-similar values presented in Quadrants II and IV. Many countries have a positive autocorrelation, while others have a negative autocorrelation, but the fitting lines indicate a positive dominant autocorrelation. The Moran I figures show that per capita CO_2_ and per capita clean energy emissions are comparable in comparable countries. In order to investigate the impact of CO_2_ emission determinants, spatial econometric models are also used.

RETRACTED

## 4. Experimental results and discussion

Two Likelihood Ratio (LR) analyses are used in this section to analyze the possibility of spatial fixed effects and time-period fixed effects being present. In two independent LR experiments, the null hypothesis is the same. It supports the model for overlapping fixed spatial and time-period effects, whereas the alternate hypothesis stresses the fixed time-period effect model and the fixed spatial effects model. The LR test statistics displayed in Table 1 display the importance of the test statistics and the dismissal of the null hypothesis for the fixed results of the time only. Therefore, the fixed spatial effects select the appropriate model to continue with the estimation process.

A couple of Lagrange Multiplier (LM) tests are also given in Table 1 to investigate whether or not the addition of spatial lag or spatial error in the model produces a substantial change in the model. For this function, autoregressive spatial error and spatially lagged dependent variable LM experiments are conducted separately using the residuals of a non-spatial model. The LM test’s null hypothesis applies to the non-spatial model, while the alternative hypothesis supports the existence of the lagging spatial model and the model of spatial error. Considering the spatial fixed effects’ presence was verified by the LR test findings, we only analyze the LM statistics for this model.

The test findings in Table 1 illustrate that the quantity of test statistics in all models is important at the level of one hundred and that spatial lag and spatial error effects need to be included in the models. Therefore, in laboratory experiments, spatial interaction effects stress the need to consider certain effects in the CO_2_ emission model.

The outcome of the Hausman test is also included in Table 2. Hypothesis null stresses the need to replace the fixed effects model with a random-effects model, while the fixed effects model bears out the alternate hypothesis. The null hypothesis is denied for all simulations, and fixed effects are verified at a 1 percent significance stage.

Finally, we test two distinct theories in Equation H_0_: θ = 0 and H_0_: θ +λβ = 0 (3). The spatial Durbin model simplifies the spatial lag model if the first theory is accepted. In comparison, the spatial Durbin model simplifies the spatial error model if the second hypothesis is accepted (Burridge [47]). The alternate hypothesis supports the independent spatial lagging variable in the model in the LR or Wald test. Both experiments have particular limitations, while Wald tests are susceptible to nonlinear restrictions, whereas LR tests need to approximate further models. So, given their ultimate outcomes and having more detailed consequences. For fixed and random-effect models, the test results in Table 3 validate the same results. On both models, the predictive significance of the LR or Wald test is important, and the spatial Durbin eventually opts for the estimation study for the spatial lagging independent.

RETRACTED

**Table 3:** The spatial Durbin model and Hausman test results.

	Model 1	Model 2	Model 3	Model 4	Model 5	Model 6	Model 7
fixed effects estimator							
Wald test: spatial Durbin model against spatial lag model	40.018	89.048	61.8	43.309	51.905	70.138	86.207
	(0.000***)	(0.000***)	(0.000***)	(0.000***)	(0.000***)	(0.000***)	(0.000***)
Wald test: spatial Durbin model against spatial error model	44.999	93.894	67.505	49.657	56.582	74.574	91.732
	(0.000***)	(0.000***)	(0.000***)	(0.000***)	(0.000***)	(0.000***)	(0.000***)
LR test: spatial Durbin model against spatial lag model	40.851	87.106	62.132	44.031	52.232	69.83	84.6
	(0.000***)	(0.000***)	(0.000***)	(0.000***)	(0.000***)	(0.000***)	(0.000***)
LR test: spatial Durbin model against spatial error model	45.643	91.431	68.194	50.172	56.958	74.586	90.877
	(0.000***)	(0.000***)	(0.000***)	(0.000***)	(0.000***)	(0.000***)	(0.000***)
random-effects estimator							
Wald test: spatial Durbin model against spatial lag model	100.371	181.378	108.325	110.753	122.613	121.653	184.673
	(0.000***)	(0.000***)	(0.000***)	(0.000***)	(0.000***)	(0.000***)	(0.000***)
Wald test: spatial Durbin model against spatial error model	76.514	150.758	82.352	90.72	93.21	94.448	136.835
	(0.000***)	(0.000***)	(0.000***)	(0.000***)	(0.000***)	(0.000***)	(0.000***)
LR test: spatial Durbin model against spatial lag model	337.192	368.04	306.91	337.197	352.931	321.729	394.015
	(0.000***)	(0.000***)	(0.000***)	(0.000***)	(0.000***)	(0.000***)	(0.000***)
LR test: spatial Durbin model against spatial error model	353.488	387.037	312.888	355.789	366.765	338.506	412.505
	(0.000***)	(0.000***)	(0.000***)	(0.000***)	(0.000***)	(0.000***)	(0.000***)
Hausman test							
Hausman test-statistic: the spatial lag model	822.546	724.346	713.493	787.561	823.803	747.305	815.587
	(0.000***)	(0.000***)	(0.000***)	(0.000***)	(0.000***)	(0.000***)	(0.000***)
Hausman test-statistic: the spatial Durbin model	69.396	819.483	43.549	51.182	32.457	66.486	170.709
	(0.000***)	(0.000***)	(0.000***)	(0.000***)	(0.006***)	(0.000***)	(0.000***)

Note: p-value, ***, **, and * show significance at 1%, 5%, and 10% level respectively.

Source: Authors’ estimations.

Table 4 indicates that most coefficients have a positive sign and a large influence on CO_2_ emissions, but clean energy efficiency and the square per capita GDP are negative. Each percent rise in per capita GDP raises emissions of CO_2_ by around 1.5%. The EKC hypothesis is confirmed, given the negative coefficient of the square term of GDP per capita. The association between GDP growth and CO_2_ emissions is an inverted U-shaped one. International direct investment has a beneficial impact on greenhouse gas emissions, which means that each unit raises CO_2_ emissions by 0.002 percent in the proportion of foreign direct investment to GDP. Urbanization also increases CO_2_ pollution, and each percent growth in urbanization raises CO_2_ emissions by around 0.4%. In addition, trade openness has also had a favorable and important impact on CO_2_ emissions, meaning that each percentage of the rise of trade openness offers the conditions for an increase in CO_2_ emissions of about 0.033 percent. In general, energy efficiency is accomplished by implementing more efficient technologies in the field of manufacturing. Energy intensity is an energy efficiency factor so that an increase in the volume of this element in the economy is equal to a reduction in energy efficiency and a deviation from technical processes. Each percentage rise in energy intensity contributes to about 0.95 percent in CO_2_ emissions, based on the data. The green energy coefficient in model 7 is pessimistic and negligible. But for clean energy elements, the findings aren’t the same. Although all 5 renewable energy elements have a negative coefficient, the results are only important for wind and solar energy. Each percent rise in solar energy contributes to a reduction in CO_2_ emissions by 0.012 percent, whereas the benefit for wind energy is 0.017.

RETRACTED

**Table 4:** The spatial lag or the spatial error in the spatial and time-period fixed effects model.

		Pooled OLS		Spatial fixed effects		Time-period fixed effects		Spatial and time-period fixed effects	
Model 1	LM spatial lag	10.607	(0.001***)	9.713	(0.002***)	12.354	(0.000***)	8.738	(0.003***)
	LM spatial error	73.668	(0.000***)	4.945	(0.026**)	71.613	(0.000***)	0.883	(0.347)
	LR-test			33.157	(0.016**)	1505.216	(0.000***)		
Model 2	LM spatial lag	10.817	(0.001***)	10.558	(0.001***)	19.583	(0.000***)	10.974	(0.001***)
	LM spatial error	77.519	(0.000***)	5.896	(0.015**)	76.176	(0.000***)	1.972	(0.16)
	LR-test			33.795	(0.013**)	1455.03	(0.000***)		
Model 3	LM spatial lag	9.855	(0.002***)	11.146	(0.001***)	12.87	(0.000***)	13.098	(0.000***)
	LM spatial error	77.77	(0.000***)	5.226	(0.022**)	75.494	(0.000***)	2.762	(0.097*)
	LR-test			46.974	(0.000***)	1517.816	(0.000***)		
Model 4	LM spatial lag	10.861	(0.001***)	11.4	(0.001***)	12.552	(0.000***)	8.662	(0.003***)
	LM spatial error	73.675	(0.000***)	5.082	(0.024**)	72.248	(0.000***)	0.902	(0.342)
	LR-test			37.088	(0.005***)	1509.438	(0.000***)		
Model 5	LM spatial lag	10.719	(0.001***)	8.278	(0.004***)	12.876	(0.000***)	9.371	(0.002***)
	LM spatial error	76.283	(0.000***)	3.6	(0.058*)	73.925	(0.000***)	1.091	(0.296)
	LR-test			32.51	(0.019**)	1499.988	(0.000***)		
Model 6	LM spatial lag	29.443	(0.000***)	8.525	(0.004***)	25.849	(0.000***)	8.671	(0.003***)
	LM spatial error	117.706	(0.000***)	3.76	(0.053*)	115.011	(0.000***)	0.839	(0.36)
	LR-test			32.535	(0.019**)	1423.254	(0.000***)		
Model 7	LM spatial lag	10.774	(0.001***)	17.198	(0.000***)	18.803	(0.000***)	19.798	(0.000***)
	LM spatial error	84.693	(0.000***)	11.108	(0.001***)	81.766	(0.000***)	8.65	(0.003***)
	LR-test			43.225	(0.001***)	1454.812	(0.000***)		

**Note**: p-value, ***, **, and * show significance at 1%, 5%, and 10% level respectively.

RETRACTED

Source: Authors’ estimations.

Heterogeneities across countries can be considered because we use spatial fixed effects. Each country gets a different intercept expression, and the key criterion for calculating the coefficients is to adjust variables over time. Term-period fixed effects also include interception over various time intervals to cover time-period heterogeneities. The elimination of such heterogeneities could boost the effects of the estimate, so it does not need to be clarified anymore, but as our diagnostic tests yield, heterogeneities are marginal and need not be considered across periods. In addition, the elimination of heterogeneities across countries means that the explanations for discrepancies across countries in terms of CO_2_ emissions are not taken into account. The coefficients in Table 5 investigate the impact of an independent variable on CO_2_ emissions over time. Therefore, if we wish to work in a cross-sectional context to understand the impact of the independent variable on CO_2_ emissions in describing the variations in CO_2_ emissions between countries, we need to use a fixed time-period effect to be the key consideration for estimating coefficients by adjusting variables over nations. In the Tables, the approximate results for the time-period fixed effects are presented (6).

**Table 5:** The estimation results for the spatial fixed effects.

	Model A1	Model A2	Model A3	Model A4	Model A5	Model A6	Model A7
*lGDPP*	2.378	2.387	2.249	2.229	2.301	2.383	2.366
	(0.000***)	(0.000***)	(0.000***)	(0.000***)	(0.000***)	(0.000***)	(0.000***)
*lGDPP* ^2^	-0.084	-0.084	-0.076	-0.073	-0.079	-0.083	-0.082
	(0.000***)	(0.000***)	(0.000***)	(0.000***)	(0.000***)	(0.000***)	(0.000***)
*FDI*	0.002	0.002	0.002	0.001	0.002	0.002	0.002
	(0.054*)	(0.039**)	(0.017**)	(0.112)	(0.023**)	(0.052*)	(0.019**)
*lURB*	0.423	0.313	0.428	0.458	0.449	0.346	0.311
	(0.000***)	(0.005***)	(0.000***)	(0.000***)	(0.000***)	(0.002***)	(0.006***)
*lOPE*	0.033	0.037	0.032	0.032	0.032	0.04	0.039
	(0.000***)	(0.000***)	(0.000***)	(0.000***)	(0.000***)	(0.000***)	(0.000***)
*lENER*	0.957	0.971	0.932	0.972	0.935	0.959	0.974
	(0.000***)	(0.000***)	(0.000***)	(0.000***)	(0.000***)	(0.000***)	(0.000***)
*lHYD*		-0.007					
		(0.613)					
*lSOL*			-0.012				
			(0.076*)				
*lWIN*				-0.017			
				(0.023**)			
*lBIO*					-0.0012		
					(0.99)		
*lGEO*						-0.03	
						(0.129)	
*lRENEW*							-0.019
							(0.161)
*W* × *lGDPP*	-0.885	-1.294	0.114	-1.098	-0.835	-0.29	-0.884
	(0.019**)	(0.000***)	(0.799)	(0.019**)	(0.026**)	(0.47)	(0.014**)
*W* × *lGDPP*^2^	0.053	0.069	-0.014	0.069	0.039	0.012	0.038
	(0.009***)	(0.000***)	(0.578)	(0.017**)	(0.06*)	(0.601)	(0.052**)
*W* × *FDI*	0	0.001	0.001	-0.001	0	-0.001	0.002
	(0.821)	(0.703)	(0.708)	(0.708)	(0.979)	(0.692)	(0.265)
*W* × *lURB*	0.575	0.39	0.26	0.661	0.574	0.681	0.271
	(0.007***)	(0.062*)	(0.254)	(0.004***)	(0.009***)	(0.002***)	(0.209)
*W* × *lOPE*	-0.107	-0.119	-0.079	-0.118	-0.096	-0.091	-0.106
	(0.001***)	(0.000***)	(0.013**)	(0.000***)	(0.003***)	(0.004***)	(0.000***)
*W* × *lENER*	0.191	0.025	0.213	0.201	0.12	0.205	-0.002
	(0.06*)	(0.803)	(0.034**)	(0.047**)	(0.238)	(0.038)	(0.987)
*W* × *lHYD*		0.237					
		(0.000***)					
*W* × *lSOL*			0.06				
			(0.000***)				
*W* × *lWIN*				-0.012			
				(0.576)			
*W* × *lBIO*					0.124		
					(0.001***)		
*W* × *lGEO*						0.257	
						(0.000***)	
*W* × *lRENEW*							0.166
							(0.000***)
*W* × *CO*_2_	0.085	0.08	0.088	0.086	0.1	0.06	0.134
	(0.141)	(0.148)	(0.126)	(0.135)	(0.079*)	(0.294)	(0.016**)

**Note**: p-value, ***, **, and * show significance at 1%, 5%, and 10% level respectively.

RETRACTED

Source: Authors’ estimations.

The results in Table 6 are the same as in Table 5, but there are several observable differences. The magnitude of the coefficients for the GDP per capita logarithm, the GDP per capita square term, trade openness and urbanization in Table 6 is somewhat larger than in Table 6, but the energy intensity coefficient is somewhat smaller. The foreign direct investment logarithm coefficient is also negligible, indicating that this variable cannot understand the explanation for the variations in CO_2_ emissions between countries. The renewable energy components show completely different results. The coefficients for hydropower, bioenergy and geothermal energy are substantially negative, indicating that lower CO_2_ emissions are produced by countries with a higher level of output of these special forms of renewable energy. Solar energy coefficients are also negative and significant, while wind energy has no significant effects. So, there is a greater amount of CO_2_ emissions in countries that produce more solar energy.

**Table 6:** The estimation results for the time-period fixed effects.

	Model B1	Model B2	Model B3	Model B4	Model B5	Model B6	Model B7
*lGDPP*	3.039	3.149	3.196	3.177	3.073	3.156	3.043
	(0.000***)	(0.000***)	(0.000***)	(0.000***)	(0.000***)	(0.000***)	(0.000***)
*lGDPP* ^2^	-0.136	-0.141	-0.146	-0.143	-0.137	-0.141	-0.135
	(0.000***)	(0.000***)	(0.000***)	(0.000***)	(0.000***)	(0.000***)	(0.000***)
*FDI*	-0.001	-0.004	-0.001	-0.001	-0.002	-0.005	-0.003
	(0.607)	(0.08*)	(0.684)	(0.562)	(0.341)	(0.027**)	(0.137)
*lURB*	0.525	0.539	0.503	0.493	0.546	0.56	0.591
	(0.000***)	(0.000***)	(0.000***)	(0.000***)	(0.000***)	(0.000***)	(0.000***)
*lOPE*	0.05	0.049	0.057	0.046	0.048	0.017	0.06
	(0.007***)	(0.006***)	(0.002***)	(0.013**)	(0.009***)	(0.319)	(0.000***)
*lENER*	0.907	0.952	0.931	0.923	0.89	0.853	0.931
	(0.000***)	(0.000***)	(0.000***)	(0.000***)	(0.000***)	(0.000***)	(0.000***)
*lHYD*		-0.061					
		(0.000***)					
*lSOL*			0.036				
			(0.04**)				
*lWIN*				-0.008			
				(0.539)			
*lBIO*					-0.062		
					(0.000***)		
*lGEO*						-0.152	
						(0.000***)	
*lRENEW*							-0.078
							(0.000***)
*W* × *lGDPP*	-0.092	0.254	-0.075	0.061	-0.147	0.311	0.3
	(0.522)	(0.057*)	(0.599)	(0.671)	(0.294)	(0.017**)	(0.022**)
*W* × *lGDPP*^2^	-0.022	-0.037	-0.022	-0.03	-0.019	-0.042	-0.041
	(0.01**)	(0.000***)	(0.011**)	(0.000***)	(0.02**)	(0.000***)	(0.000***)
*W* × *FDI*	-0.006	-0.01	-0.005	-0.007	0.002	-0.008	-0.007
	(0.304)	(0.091*)	(0.409)	(0.231)	(0.751)	(0.157)	(0.201)
*W* × *lURB*	0.625	0.143	0.673	0.565	0.78	0.21	0.172
	(0.000***)	(0.327)	(0.000***)	(0.000***)	(0.000***)	(0.118)	(0.224)
*W* × *lOPE*	0.04	0.07	-0.012	-0.012	0.012	-0.071	0.053
	(0.497)	(0.206)	(0.848)	(0.845)	(0.836)	(0.197)	(0.328)
*W* × *lENER*	-0.219	-0.323	-0.254	-0.313	-0.277	-0.163	-0.383
	(0.02**)	(0.000***)	(0.007***)	(0.001***)	(0.003***)	(0.055*)	(0.000***)
*W* × *lHYD*		-0.007					
		(0.746)					
*W* × *lSOL*			-0.066				
			(0.049**)				
*W* × *lWIN*				-0.09			
				(0.002***)			
*W* × *lBIO*					-0.108		
					(0.003***)		
*W* × *lGEO*						0.016	
						(0.719)	
*W* × *lRENEW*							-0.009
							(0.69)
*W* × *CO*_2_	0.139	0.246	0.123	0.167	0.114	0.256	0.249
	(0.001***)	(0.000***)	(0.003***)	(0.000***)	(0.005***)	(0.000***)	(0.000***)

**Note**: p-value, ***, **, and * show significance at 1%, 5%, and 10% level respectively.

Source: Authors’ estimations.

Spatial models enable the direct and indirect effects of independent variables to be separated. Direct effects measure the effect of the independent variable on the spatially dependent variable, while indirect effects measure the effect of the independent variable on the spatially dependent variable of the neighboring region. The actual and indirect effects of the independent variables in Model 2 and the clean energy variables in Models 3 to 6 are shown in Table 7. The direct effects differ slightly from the parameter estimated in Table 5 because feedback effects resulting from the impact of crossing neighboring countries and returning to the countries themselves are included in the direct effects.

RETRACTED

**Table 7:** Marginal effects of the CO_2_ emission determinants.

	Direct		Indirect		Total	
	Coefficient	p-value	Coefficient	p-value	Coefficient	p-value
*lGDPP*	2.357	(0.000***)	-0.742	(0.06*)	1.615	(0.001***)
*lGDPP* ^2^	-0.082	(0.000***)	0.05	(0.027**)	-0.033	(0.21)
*FDI*	0.002	(0.067*)	0	(0.847)	0.001	(0.602)
*lURB*	0.439	(0.001***)	0.664	(0.01**)	1.102	(0.002***)
*lOPE*	0.032	(0.001***)	-0.111	(0.003***)	-0.079	(0.041**)
*lENER*	0.96	(0.000***)	0.293	(0.003***)	1.253	(0.000***)
*lHYD*	-0.003	(0.843)	0.253	(0.000***)	0.251	(0.000***)
*lSOL*	-0.011	(0.115)	0.063	(0.000***)	0.052	(0.004***)
*lWIN*	-0.018	(0.022**)	-0.016	(0.536)	-0.033	(0.232)
*lBIO*	0.003	(0.82)	0.138	(0.002***)	0.142	(0.006***)
*lGEO*	-0.026	(0.188)	0.267	(0.000***)	0.241	(0.000***)
*lRENEW*	-0.014	(0.283)	0.186	(0.000***)	0.171	(0.000***)

**Note:** p-value, ***, **, and * show significance at 1%, 5%, and 10% level respectively.

Source: Authors’ estimations.

The findings show that neighboring countries’ economic growth and trade access negatively impact countries’ domestic CO_2_ emissions. Every percent rise in neighboring countries’ economic growth contributes to reducing domestic CO_2_ emissions by 0.742 percent. This value is 0.111 for economic transparency. There is also a positive influence on domestic CO_2_ pollution from the urbanization of neighboring countries. The findings suggest that increased renewable energy production in neighboring countries contributes to higher domestic CO_2_ emissions. For wind power alone, the coefficient is not important.

## 5. Conclusion and policy implications

From 2000 to 2018, this analysis used evidence from 31 Asia-Pacific countries to analyze the impact of a few independent variables on CO_2_ emissions, while the effects of renewable energy components are highlighted in more detail. The diagnostic assessments assess the Durbin spatial model such that the spatial relationship practically has to be taken into account in the CO_2_ emission model. As a consequence of the eliminated component, the lack of consideration of the spatial effects in the scientific literature contributes to the skewed calculation, so spatial econometrics in the CO_2_ emission model is a must.

RETRACTED

The test findings demonstrate that most independent variables, including GDP per capita, openness to trade, urbanization, and electricity intensity, substantially positively affect CO_2_ emissions. The EKC hypothesis is confirmed, and there is an inverted U-shaped impact of GDP per capita on CO_2_ emissions. The findings suggest that the growth of the manufacturing sector and trade openness in neighboring countries will decrease domestic CO_2_ emissions, possibly because the expansion of regional competitiveness will impact the domestic manufacturing sector and reduce emissions. Moreover, higher energy intensity will contribute to increased CO_2_ pollution in neighboring countries. Also, the production of renewable energy in nearby countries produces the same results. The performance of the results is very fair, unlike the obvious disparity in the spatial fixed effects results and the time-period fixed effects models for renewable energy sources. Since solar and wind power categories the countries under review as newer types of renewable energy, the shares of these two particular types of overall renewable energy in 2000 were around 0.07 percent and 0.24 percent, respectively, while the shares rose to 15.6 percent and 8.6 percent in 2018. The share of hydropower electricity has decreased from around 94.7 percent to 69.9 percent during this time. Over time, the other forms have similar shares. According to the findings of the Spatial Fixed Effects Model, the growth of and substitution of solar and wind resources instead of hydropower has, over time, contributed to a decrease in air emissions in countries.

On the other hand, the time-period model of fixed effects reveals that more solar energy is generated in other older renewable energy sources, such as hydropower, bioenergy and renewable energy, which are produced in countries with higher levels of CO_2_ emissions. In countries with lower levels of CO_2_ emissions, geothermal energy levels are higher. These findings show that air pollution in countries with higher levels of CO_2_ emissions is more prevalent. These findings show that countries need more foresight and focus in pushing toward solar and wind clean energy, so achieving a high level of emissions cannot be a catalyst in this direction, and mitigation is a more successful path.
